# Separation of Different Blogs from Skin Disease Data using Artificial Intelligence

**DOI:** 10.1155/2022/7538643

**Published:** 2022-08-23

**Authors:** Mohammed J. Abdulaal, Ibrahim M. Mehedi, Abdulah Jeza Aljohani, Ahmad H. Milyani, Mohamed Mahmoud, Abdullah M. Abusorrah, Rahtul Jannat

**Affiliations:** ^1^Department of Electrical and Computer Engineering (ECE), King Abdulaziz University, Jeddah, Saudi Arabia; ^2^Center of Excellence in Intelligent Engineering Systems (CEIES), King Abdulaziz University, Jeddah, Saudi Arabia; ^3^Electrical and Engineering Department, Tennessee Technological University, Cookeville, TN, USA; ^4^Department of Electrical and Electronic Engineering, BRAC University, Dhaka, Bangladesh

## Abstract

A combination of environmental conditions may cause skin illness everywhere on the earth, and it is one of the most dangerous diseases that can develop as a result. A major goal in the selection of characteristics is to produce predictions about skin disease instances in connection with influencing variables, which is one of the most important tasks. As a consequence of the widespread usage of sensors, the amount of data collected in the health industry is disproportionately large when compared to data collected in other sectors. In the past, researchers have used a variety of machine learning algorithms to determine the relationship between illnesses and other disorders. Forecasting is a procedure that involves many steps, the most important of which are the preprocessing of any scenario and the selection of forecasting features. A major disadvantage of doing business in the health industry is a lack of data availability, which is particularly problematic when data is provided in an unstructured format. Filling in missing numbers and converting between various types of data take somewhat more than 70% of the total time. When dealing with missing data in machine learning applications, the mean, average, and median, as well as the stand mechanism, may all be employed to solve the problem. Previous research has shown that the characteristics chosen for a model's overall performance may have an influence on the overall performance of the model's overall performance. One of the primary goals of this study is to develop an intelligent algorithm for identifying relevant traits in models while simultaneously eliminating nonsignificant attributes that have an impact on model performance. To present a full view of the data, artificial intelligence techniques such as SVM, decision tree, and logistic regression models were used in conjunction with three separate feature combination methodologies, each of which was developed independently. As a consequence of this, their accuracy, *F*-measure, and precision are all raised by a factor of ten, respectively. We then have a list of the most important features, together with the weights that have been allocated to each of them.

## 1. Introduction

Both climate change and global warming are well-known phenomena, and climate change is a process that has been going on for a long period of time. In the atmosphere of the planet, a mixture of inward-directed solar radiation and outward-directed thermal radiation is responsible for maintaining its temperature. There are a variety of factors that contribute to global climate change and the warming of the Earth's atmosphere. Some of these factors include greenhouse gases, radiation, carbon dioxide, wind patterns, methane, fossil fuel emissions, ocean currents, and other factors. In recent years, carbon dioxide emissions from fossil fuels have increased, and some research suggests that population expansion may be one of the most important contributors to this trend [1]. There has been a published study on this issue by [2]; environmental scientists have said in previous studies that the change in climate has substantially risen over the past few years, according to the environmental science collective. In the future, according to the IPCC, CO_2_ concentrations will rise to [3] 300–400 parts per million (ppm), with an associated increase in ocean acidity of 25% and an increase in the global average temperature of between 0.18 and 0.22°C [4]. According to previous studies, the majority of infectious diseases, such as dengue, Zika, chikungunya, malaria, heart disease, and skin disease, are on the increase. When doing our research, we sought incidences of skin sickness that were associated with environmental factors such as climate [5]. Solar ultraviolet (UV) radiation inflicts direct damage to both the inner and exterior pigments of the cell, leading to a range of skin disorders, including sunburn [6].

Dermatological problems are very susceptible in the presence of extended exposure to UV light. It is possible that this is due to the age distribution in the data set; according to the study, men between the ages of 30 and 45 are at higher risk than females in the same age range, which may explain why [7]. Moreover probable is death as a consequence of the negative influence of climatic conditions on one's mental well-being. The International Classification of Disorders and the Intergovernmental Panel on Climate Change estimate that illness is responsible for 30% of all skin disorders reported to the medical community [8]. Compared to other infectious diseases, skin disorders are caused by burns on the body's surface and are only marginally less dangerous in terms of prevention and control when compared to other infectious diseases [9]. Abscesses, enzymes, fungal infections, psoriasis, acne vulgaris, urticaria, alopecia areata, priority, and deceits ulcers are some of the subcategories of skin diseases that may be classified. The topic was addressed by a great number of authors in previous studies, who used both traditional and analytical approaches to try to solve it [10]. The machine learning model that is used in the analysis of health-care data is called a deep learning model. Several algorithms have been developed to detect diseases in real time while taking medical data into consideration and predicting any symptoms that may arise [11].

No matter how many missing values and hidden patterns there are in real-time medical data, each piece of information must be properly preprocessed and picked before the disease diagnosis process can begin in earnest [12]. There is no ready-to-use medical data; instead, we must fill in the blanks, convert the constant value to a categorical variable, and rename the columns to get a rudimentary understanding of the information contained inside them. If you are having trouble filling in the blanks, one of the first steps you should do is to utilize the machine learning mean and the average of the missing column, which are solid strategies that may be employed to help [13]. The type dialogue method is used to convert continuous values to absolute values (and vice versa), and the column change function is used to modify the name of the column in question. We have determined that the data set is ready for analysis after all the aforementioned steps have been completed; nevertheless, we have determined that the following phases are more critical and harder to perform. In part because of the enormous number of attributes included in medical data, it is possible that even the most illogical traits may have an influence on the model's performance [14]. In machine learning models, a particular procedure called feature selection is used to pick the features that will be included in the model. This study will solely use a supervised feature selection technique due to the fact that our data has been supervised so far. A combination technique is being used in this research to (1) preprocess the raw data and (2) choose meaningful features from the raw data.

Literature is number two on the list. Through the use of feature selection approaches, the author hopes to develop a new classification system. Prior to going on to further investigations, further study would often start with feature selection, followed by rating, before moving on to additional inquiries. According to the documentation, the model's execution time was rather lengthy. After initially categorizing the feature set, the genetic algorithm that has been proposed picks the feature set from among the classes [15]. Artificial immune systems have a higher number of properties than natural immune systems. The authors propose a filter selection mechanism that is based on the geographic location of the user. The proposed approach looks for samples of adjacent neighbors who are related to one another to find them [16]. Antimicrobial resistance is a large public health problem all throughout the globe, particularly in developing countries. According to the authors, a time series method for disease outbreak prediction may be utilized to directly anticipate the commencement of disease epidemics. They use the wrapper approach as a component of their feature selection strategy [16]. In most cases, cardiovascular disease analysis is a crucial stage in which the authors seek to predict in a short amount of time utilizing just the most impactful attribute. It is proposed by the authors to use a hybrid feature selection strategy that incorporates a combination of two to three models [17]. Medical data collection for TCM disorders is predicted to include 200 features, according to the researchers. If you are trying to reduce or eliminate irrelative quality, the authors recommend that you use the ANN feature selection approach to do so [18]. Clinical data are becoming more common in all health departments, and access to such data is entirely unrestricted in the unstructured text format. The authors wrote their work using the dictionary-based strategy, which he developed himself. When dealing with static data, unnecessarily complicated situations are more common [19]. The authors suggested that attributes be selected from a limited selection of possibilities. Missing values and other data difficulties are dealt with using a mixed technique in this case. Due to the fact that medical data is easily available and is created in vast amounts, this is the situation. When dealing with missing value data, the authors suggested a two-step technique (1) to compress high-dimensional data and (2) to differentiate between distinct categories and numeric value data when dealing with missing value data. Typically, since labelling is done one at a time, the multilabel selection problem is one that is difficult to resolve. The authors advised that features be selected in a discriminating and relevant manner, among other things. The authors recommended employing the variance feature section approach for gene selection in their paper [20].

## 2. Data Collection and Methods

The Ontario General Hospital is a vibrant institution that is always crowded with patients suffering from a broad variety of diseases and ailments. On average, the hospital handles between 6,000 and 8,000 patients every day, with many of them being treated in a variety of departments around the institution, according to the in-patient statistics. According to the dermatology department, patients with skin-related disorders make between 150 and 200 visits every week to the department, depending on the severity of their condition. In regard to dermatology, the number of patients visiting the department is growing at the same time as the overall temperature is rising. Patients at the OGH hospital who were undergoing skin-related treatment as a result of the change in the environment provided us with the information we needed for our study. According to the India Meteorological Department (IMD), in this situation, the data set collected from the IMD is based on the city limits of Hyderabad, which falls under the jurisdiction of the IMD Zone 4 weather forecasting division. Throughout the data set, there are daily and monthly observations for the variables, which span the years 1995–2018. From 1995 to 2018, the data set contains data for the variables temperature, precipitation, rainfall, humidity, and precipitation, as well as other variables as shown in Table 1. It took two phases to complete this research; in the first phase, data from the hospital were collected, and tests were carried out, and in the second phase, data were collected, and further experiments were conducted. As a result of receiving climate data collected from the National Data Centre of India, we have officially entered our second phase (India Meteorological Department). Specific to this study is a determination of the relationship between meteorological data and hospital data. Males and females have been allocated the numbers 0 and 1, respectively, in this study to distinguish between them. According to the experimental data, which we obtained from the research's outcomes, males were more adversely impacted than women in the study. Females are exposed to light for a shorter period of time than men, according to the researchers, and this is the basis for their discovery. We have created a graph based on the data, and it is clear that 67.2% of males and 32.8% of women suffer from a skin condition as shown in Figure 1.

To overcome this problem, we have presented a framework as shown in Figure 2. The suggested framework is a mix of trial and error and data-driven techniques. There are a total of 20 characteristics in the data set with 1,500 occurrences, which were verified using the model before and after.

### 2.1. Preprocessing

Since 2014, there has been a considerable growth in the volume of data produced. The term “data set” refers to a variety of various sorts of information, including movies, structures, sounds, and photographs, among other things. The data format should be machine-readable, that is, consisting only of 0's and 1's, since a computer will be unable to grasp the data format if it is not. Preprocessing is a single step in the machine learning mechanism that helps a computer comprehend what it is learning. It is performed before the computer begins to learn. The data set is made up of a range of pieces, including a sample, entity, points, occurrences, patterns, and observations, among others. It is a data object that contains the number of attributes or variables included in a data item; data are classified into two types: categorical and numerical, as shown in Figure 3.

Due to the fact that the data obtained from diverse sources are raw data, the quality of data stored by applying the preprocessing approach might have an impact on the accuracy of the model.

(1) Find the local extrema of the signal by identifying the change of sign of the derivative of the signal, *s*(*t*)
(2) Construct two splines that connect all minima and maxima of the signal to identify the upper and lower envelopes
(3) Find the first component, *h*_1_, from the two envelopes, given by the following equation:
  (1) $$\begin{array}{c} s\left(t\right)-m_{1}=h_{1}, \end{array}$$

where *m*_1_ is the mean of the envelopes. This is called first round shifting. Here, *h*_1_ is referred as proto-IMF. In the second round, it is treated as a signal.

(2) $$\begin{array}{c} h_{1}-m_{11}=h_{11}. \end{array}$$

After repeatedly shifting *k*-times, *h*_1*k*_ is obtained, which is given by the following expression:

(3) $$\begin{array}{c} h_{1\left(k-1\right)}-m_{11}=h_{1k}, \end{array}$$

The function *h*_1*k*_ is known as the first IMF component, given by

(4) $$\begin{array}{c} c_{1}=h_{1k}. \end{array}$$

1. Stop the shifting process when the stopping criteria, SD_*k*_, is smaller than a predefined value.
  (5) $$\begin{array}{c} SD_{k}=\frac{\sum_{t=0}^{T}{\left|h_{k-1}\left(t\right)-h_{k}\left(t\right)\right|}^{2}}{\sum_{t=0}^{T}h_{k-1}^{2}\left(t\right)}. \end{array}$$
(2) Find the residue of the signal using the following equation:
  (6) $$\begin{array}{c} s\left(t\right)-c_{1}=r_{1}. \end{array}$$

Repeat the process for all the values of *r*_*j*_ and obtain the results using the following equations:

(7) $$\begin{array}{c} r_{1}-c_{2}=r_{2},\\ r_{n-1}-c_{n}=r_{n}. \end{array}$$

The above process is stopped, when the residue, *r*_*n*_, is changed into a monotonic function. The original signal *s*(*t*) is obtained by summing the above equations.

(8) $$\begin{array}{c} s\left(t\right)=\sum_{j=1}^{n}c_{j}+r_{n}. \end{array}$$

The instantaneous frequency of the signal is calculated by finding the Hilbert transform of the IMFs. The original signal is represented as the real part of RP using the following equation:

(9) $$\begin{array}{c} s\left(t\right)=RP\left\{\sum_{j=1}^{n}a_{j}\left(t\right)e^{i\int w_{j}\left(t\right)dt}\right\}. \end{array}$$

The signal *s*(*t*) is expressed in terms of the Fourier series, as follows:

(10) $$\begin{array}{c} s\left(t\right)=RP\left\{\sum_{j=1}^{\infty }a_{j}e^{iw_{j}t}\right\}. \end{array}$$

It results in missing gaps during data collection, which may be caused by a machine or human error at the moment of recording. There are a few solutions, such as removing rows and columns, but they will be ineffective since they lessen the sensitivity of the data.

### 2.2. Input Feature Sets

Due to the fact that medical data contains the irrelative quality that may have an impact on model performance, not all attributes are relevant. The number of features in a model always changes the model and makes it more complicated. Aims of any feature selection strategy include improving model performance, providing a cost-effective and speedier comprehension of the underlying patterns, and reducing model complexity. There are three different sorts of strategies for feature selection as shown in Figure 4.

According to the score variables that have been picked, it ranks fitter approach is used by a statistical methodology to award a score to each variable. Wrapper method: choosing features from a variety of feature combinations and comparing them to other feature combinations is performed. To decrease the coefficients to zero, ensemble methods such as the regularization approach and penalization of the data are used.

### 2.3. Machine Learning Model

After taking into account all factors, we used three machine learning techniques for the analysis: the support vector machine (SVM), decision tree, and logistic regression. The tenfolds approach is used for model validation, and then the data are separated into ten subgroups, which is a procedure that is repeated ten times. It makes use of one subset of data for training and nine further subsets of data for testing. Following that, the average of ten iterations is shown. The stratified approach is used to divide the data set into two groups.

### 2.4. Model Performance

The precision, accuracy, and *F*–measure [21–23] of machine learning algorithms are statically tested to determine their performance. These three performance measures were utilized to choose important characteristics; in general, most machine learning models use one or more performance metrics to identify significant features. Performance measurements are quite important in the selection of several qualities, and they play an important part in this [24–29]. It is necessary to use a different combination set of variable. The overarching concept is to eliminate irrelative features that are interfering with the performance of the model. In the following tables, you can find the results of all three metrics' performance calculations and records.

(11) $$\begin{array}{c} \mathrm{Accuracy}=\frac{\left(\mathrm{TP}+\mathrm{TN}\right)}{\left(\mathrm{TP}+\mathrm{TN}+\mathrm{FP}+\mathrm{FN}\right)},\\ \text{F}-\text{Measure}=\frac{\left(2*\mathrm{Precision}*\mathrm{Recall}\right)\;}{\;\left(\mathrm{Precision}+\mathrm{Recall}\right)},\\ \mathrm{Precision}=\frac{\mathrm{True}\;\mathrm{Positives}}{\left(\mathrm{True}\;\mathrm{Positives+False}\;\mathrm{Positives}\right)}. \end{array}$$

## 3. Results

Hidden patterns were discovered in our data set, which had 20 characteristics with 1,500 occurrences, and we utilized 3 different machine learning techniques to uncover them. By picking a set of qualities utilizing a machine learning pipeline and performance measurements, we are employing a trial-and-error combination strategy to conduct our experiments. Model validation is accomplished using *F*-measure, precision, and accuracy. Following the data analysis, we provide the greatest accuracy, highest precision, and highest *F*-measure in Tables 2–4. When compared with other algorithms in Table 2, the three tables below show three distinct machine method models with 11 characteristics using SVM with excellent accuracy. While the decision tree gets a high accuracy rate by using a variety of combination tables, the SVM fared very well in the *F*-measure when compared to other models. In regard to predicting, the mix of several factors is quite important.

The major feature selection has been accomplished by the application of the techniques described above, and in the table below, each attribute count is recorded in three separate performance metrics. During the final stages of a feature, the incidence rate of counts is shown. Depending on the number of components, they are rated and assigned a relative priority, which aids in better predicting [18]. The significant factors are further analyzed to anticipate the incidence of skin disease by combining the significant variables in a new manner. Our experiment demonstrates that increasing the number of features in a certain variable and applying machine learning models with their corresponding performance metrics to a list of feature importance leads to an increase in the number of features. With the aid of the Python programming language, the scikit-learn pipeline is used to analyze the model and choose features. The performance of the machine learning model is verified by taking into account the feature pre- and postdata [6]. When comparing the accuracy rates before and after feature selection, it is clear that the accuracy rate is much lower before feature selection and significantly higher after feature selection.

## 4. Discussion

Algorithms for machine learning with varied combinations of data sets, SVM, decision tree, and logistic regression were used to try to uncover a meaningful variable [19]. The accuracy of the algorithm is shown both with and without feature selection. The final accuracy result demonstrates that the accuracy rate has increased as a consequence of the addition of a new feature set. These characteristics are expected to make a major contribution to the forecasting of skin disorders connected with environmental variables. IMD collects 16 climatic characteristics out of a total of 20 factors; the gender of patient attributes is connected to demographic information. After conducting a thorough investigation, we discovered that the peculiarities of climatic conditions had a greater impact on skin problems. According to our findings, the suggested framework obtained an 84% success rate with the bare minimum of features as shown in Tables 5 and 6.

These discoveries have prompted the exploration of a new research gap, which has resulted in the use of various preprocessing and feature selection strategies. Both steps are more crucial in data analysis, with cleaning and feature selection accounting for roughly 70% of the total time spent on the task. Our full feature set will be released soon. The suggested framework aids in the investigation of disease outbreaks. Our research demonstrates that by using tail and error combination accuracy, we were able to get excellent accuracy, which was then confirmed using performance measures such as accuracy, *F*-measure, and precision.

## 5. Conclusion

An exponential increase in the amount of data generated by the sector has happened during the last few years. The health business has seen one of the most substantial surges in data creation in recent history. Everything acquired by the preinstalled sensor, regardless of how good the data is in terms of quality, is stored in a raw format that cannot be manipulated. Machine learning technologies are used to fulfil the tasks of preprocessing and feature selection in this study. Unformatted unsigned values are present in the data set, and the machine is unable to read them because they are incompatible with the machine's ability to read them. The time spent on preprocessing and feature selection accounted for more than 70% of the overall time spent. It is possible to anticipate the emergence of any ailment by taking into consideration the most important factor, making the data publicly accessible, and presenting it in an easily understandable manner. To do this, we integrated three independent machine learning models, each with a unique set of attributes, into a single model. For verifying the model's performance, three performance matrices have been used to assess its performance. When compared to other models, the SVM model has the highest accuracy, with an accuracy of 84% when employing the new feature set, according to the new feature set. Our data set is unique in that it is the only benchmark data accessible; thus, we have not compared it to any other study that has been undertaken. In our investigation, one of the major flaws was the absence of any dimensionality reduction techniques. This necessitates the use of stranded preprocessing and feature selection techniques. There is always a limit to the amount of data that may be collected in each research effort.

## Figures and Tables

**Figure 1:** Male versus female gender ratio.

**Figure 2:** Proposed framework.

**Figure 3:** List of data types is the data set in supervised learning.

**Figure 4:** Types of feature selection techniques.

**Table 1:** Representation of all feature names with data types.

Number	Features	Type	New_feature_name
1	Total precipitation	Float64	*F*11
2	Southeast_NDVI	Float64	*F*12
3	Max_air_temp	Float64	*F*13
4	Total_precipitation in KG	Float64	*F*14
5	Northeast_NVDI	Float64	*F*15
6	Diurnal_temp	Float64	*F*16
7	Northwest_NDVI	Float64	*F*17
8	Mean_duepoint	Float64	*F*18
9	South_NDVI	Float64	*F*19
10	Mean humidity	Float64	*F*20

**Table 2:** SVM versus decision tree versus logistic regression with the feature set.

Models	Precision (%)	Features_set
SVM	75.03	Features −1, 3, 5,7, 9, 11, 13, 15, 17, 19
Decision tree	**84.12**	Features −1, 2, 5, 9, 11, 13, 17, 8
Logistic regression	74.90	Features −1, 2, 4, 6, 8, 10, 12, 14, 16, 18, 20

**Table 3:** SVM versus decision tree versus logistic regression with the feature set.

Models	*F*-measure (%)	Features_set
SVM	**83.32**	Features −1, 3, 5, 7, 9, 11, 13, 15, 17, 19
Decision tree	81.45	Features −1, 2, 5, 9, 11, 13, 17, 8
Logistic regression	82.75	Features −1, 2, 4, 6, 8, 10, 12, 14, 16, 18, 20

**Table 4:** SVM versus decision tree versus logistic regression with the feature set.

Models	Accuracy (%)	Features_set
SVM	**84**	Features −1, 3, 5, 7, 9, 11, 13, 15, 17, 19
Decision tree	80	Features −1, 2, 5, 9, 11, 13, 17, 8
Logistic regression	81	Features −1, 2, 4, 6, 8, 10, 12, 14, 16, 18, 20

**Table 5:** Final model accuracy with the old and new feature sets.

Final accuracy	SVM (%)	Decision tree (%)	Logistic regression (%)
With all features (20)	83.12	81.74	79.63
With new features (11)	84	82.87	80.32

**Table 6:** List of feature importance weights.

Number	Features	New_feature_name	Feature_weights
1	Year_week	*F*1	0.0899
2	Recorded_year	*F*2	0.0612
3	Recorded_month	*F*3	0.0394
4	Air_temp	*F*4	0.0174
5	Humidity	*F*5	0.0167
6	Surface_water3	*F*6	0.0152
7	Total_vegetation	*F*7	0.0101
8	Min_air_temp	*F*8	0.0069
9	Surface_water5	*F*9	0.0058
10	Surface_water1	*F*10	0.0051
11	Total_precipitation	*F*11	0.0013
12	Southeast_NDVI	*F*12	0.003
13	Max_air_temp	*F*13	0.0003
14	Total_precipitaion in KG	*F*14	0.0002
15	Northeast_NVDI	*F*15	0
16	Diurnal_temp	*F*16	−0.0002
17	Northwest_NDVI	*F*17	−0.0019
18	Mean_duepoint	*F*18	−0.0046
19	South_NDVI	*F*19	−0.0054
20	Mean_humidity	*F*20	−0.0067

## Data Availability

This article contains all the data used to support this study.
